# Angiotensin II Mediates Cardiomyocyte Hypertrophy in Atrial Cardiomyopathy via Epigenetic Transcriptional Regulation

**DOI:** 10.1155/2022/6312100

**Published:** 2022-06-17

**Authors:** Liuying Zheng, Jin Wang, Rui Zhang, Yingyi Zhang, Jie Geng, Lu Cao, Xiaoyun Zhao, Jianhui Geng, Xinping Du, Yuecheng Hu, Hongliang Cong

**Affiliations:** ^1^Tianjin Medical University, Heping District, Tianjin 300070, China; ^2^Department of Cardiology, Tianjin Chest Hospital, Jinnan District, Tianjin 300222, China; ^3^Cardiac Surgery, Peking University First Hospital, Xicheng District, Beijing 100034, China; ^4^Department of Respiratory Critical Care Medicine and Sleep Center, Tianjin Chest Hospital, Tianjin 300222, China; ^5^Tianjin University, Tianjin 300072, China; ^6^Tianjin Tiangong University, Life Science School, Tianjin 300387, China; ^7^Shanxi Cardiovascular Hospital, 18 Yifen Street, Taiyuan, 030024 Shanxi, China; ^8^Department of Cardiology, The Fifth Central Hospital of Tianjin, Binhai Hospital of Peking University, Binhai New Area, Tianjin 300450, China

## Abstract

**Aims:**

European Heart Rhythm Association established an expert consensus to define, characterize, and classify atrial cardiomyopathy into four subgroups based on their histopathological features. The predominant pathological feature of classes I and III is the hypertrophy of atrial cardiomyocytes. Here, we aim to investigate the mechanism of epigenetic transcriptional regulation of cardiomyocyte hypertrophy in atrial cardiomyopathy.

**Methods and Results:**

Compared with that of sinus rhythm control individuals, the myocardium of patients with atrial fibrillation exhibited increased levels of angiotensin II (AngII), chromatin-bound myocyte enhancer factor 2 (MEF2), acetylated histone H4 (H4ac), and H3K27ac; upregulation of hypertrophy-related genes; and decreased levels of histone deacetylase (HDAC) 4 and HDAC5 bound to the promoters of hypertrophy-related genes. Furthermore, incubation of atrial cardiomyocytes with AngII increased their cross-sectional area and improved the expression of hypertrophy-related genes. AngII also promoted the phosphorylation of HDAC4 and HDAC5 and induced their nuclear export. RNA sequencing analyses revealed that AngII significantly upregulated genes associated with cardiac hypertrophy. Chromatin immunoprecipitation showed that this correlated with increased levels of chromatin-bound MEF2, H4ac, and H3K27ac and decreased HDAC4 and HDAC5 enrichment in the promoters of hypertrophy-related genes. Moreover, these AngII-induced prohypertrophic effects could be partially reverted by treatment with the AngII receptor blocker losartan.

**Conclusions:**

AngII had a prohypertrophic effect on atrial cardiomyopathy which was epigenetic-dependent. Patients with atrial fibrillation manifest an increased susceptibility to hypertrophy and exhibit epigenetic characteristics that are permissive for the transcription of hypertrophy-related genes. AngII induces histone acetylation via the cytoplasmic-nuclear shuttling of HDACs, which constitutes a novel mechanism of atrial hypertrophy regulation and might provide a promising therapeutic strategy for atrial cardiomyopathy.

## 1. Introduction

From the first observation as “auricle” by Harvey [1] in 1628 to the latest definition as “atrial failure” by Bisbal et al. [2] in 2020, we went through a nearly 400-year journey of atrial study. The evolution of the atrial pathophysiological terms has experienced “atrial remodelling” [3], “atrial fibrillation(AF)” [4], “atrial cardiomyopathy” [5], “atrial dysfunction” [2], etc. AF constitutes the most commonly encountered arrhythmia in clinical practice and a major cause of mortality [4]. Structural remodelling is the main contributing mechanism and hallmark of AF [2, 3], and we have shown that stress-induced atrial structural remodelling in particular plays an important role in AF progression [6, 7]. In 2016, the European Heart Rhythm Association and four other associations define, characterize, and classify atrial cardiomyopathy into four subgroups based on their histopathological features [5]. The working group proposed the following working definition of atrial cardiomyopathy: “Any complex of structural, architectural, contractile, or electrophysiological changes affecting the atria with the potential to produce clinically relevant manifestations” [5], emphasizing the close correlation among structural, electrophysiological, and functional remodelling in atrial pathogenic substrates. However, the mechanisms underlying atrial cardiomyopathy initiation and progression have not been systematically delineated. Better understanding of atrial cardiomyopathy pathogenesis may foster breakthroughs in the therapeutic treatment of atrial dysfunction, AF, and cardiogenic stroke.

The predominant pathological feature of class I and III atrial cardiomyopathy is atrial cardiomyocyte hypertrophy [5]. Cardiomyocytes are terminally differentiated and lose their capacity to proliferate soon after birth. Thereafter, cardiomyocytes grow in size without cell proliferation to adapt to the demand for overload. In several pathological conditions (e.g., hypertension, valvular disease, and myocardial infarction) that impose overwork on the heart, postnatal cardiomyocytes undergo cardiac hypertrophy. Although initially compensatory for overload, prolongation of this stressed process leads to congestive heart failure, arrhythmia, and sudden death [8]. At the cellular level, cardiac hypertrophy is characterized by an increase in cell size and reactivation of the foetal gene program [9].

Angiotensin II (AngII) is a major effector peptide in angiotensin system (RAS), which usually stimulates hypertrophy [10]. Hypertrophic stimuli initiate a number of subcellular signalling pathways that eventually lead to altered cardiac myocyte gene expression via transcription factors including myocyte enhancing factor-2 (MEF2) [11] and a zinc finger protein, GATA-4 [12]. Increasing evidence also suggests that epigenetic mechanisms are involved in RAS-induced cardiac remodelling [13]. Epigenetic regulation such as histone (H3 and H4) lysine acetylation (H3Kac and H4Kac) plays an important role in gene transcription regulation, while histone deacetylase (HDAC) promotes chromatin structural condensation, leading to transcriptional suppression [14, 15].

Transcription factor MEF2 associates with class II HDACs via an 18-amino-acid motif [16, 17]. Class II HDACs form a complex with MEF2 via gene regulatory elements, resulting in repression of genes transcription by harbouring MEF2-binding sites [18]. HDACs shuttled from the nucleus to the cytoplasm in response to stress, providing an epigenetic mechanism to override HDAC-mediated repression of cardiac growth [19]. This redistribution of HDACs enables MEF2 and other transcriptional activators to associate with histone acetyltransferase (HAT) [20] resulting in increased local histone acetylation and activation of downstream genes that facilitate cellular growth.

However, the nuclear transcriptional mechanism of AngII signalling as well as the potential involvement of epigenetic chromatin remodelling in cardiac hypertrophy remain unexplored. In the present study, we showed that atrial samples from patients with AF displayed increased susceptibility to hypertrophy and epigenetic characteristics that are permissive for hypertrophy-related gene transcription. In primary neonatal cardiomyocytes, we showed that by inducing cytoplasm nuclear shuttling of HDACs, AngII regulates histone acetylation, promoting MEF2 binding to the promoter of hypertrophy-related genes and representing a novel mechanism for atrial hypertrophy.

## 2. Methods

### 2.1. Experimental design

Animal care and isolation procedures were approved by the Animal Ethics Committee of the 5th Central Hospital of Tianjin, China, and were performed according to the European Directive on Laboratory Animals (86/609/EEC). All experimental procedures were performed according to the Guide for the Care and Use of Laboratory Animals (NIH Publication No. 85-23, revised 1996) and were in compliance with the guidelines specified by the Chinese Heart Association policy on the use of research animals and the Public Health Service policy on the use of laboratory animals.

### 2.2. Human Atrial Samples

Consecutive patients with valvular heart disease who underwent mitral or aortic valve replacement or coronary artery bypass grafting were recruited. Patients taking angiotensin converting enzyme inhibitors and/or angiotensin II-receptor blockers (ARBs) were excluded from the study. Overall, a total of eight patients with chronic persistent atrial fibrillation (AF group) and seven patients without a history of AF (sinus rhythm, SR group) were recruited. All patients underwent echocardiography before the surgery. Samples of right atrial appendages were obtained during open-heart surgery, quickly frozen in liquid nitrogen, and maintained at −80°C until used for mRNA and protein analysis. The study protocol was approved by the Ethics Committee of 5th Central Hospital of Tianjin, China. The research protocol was registered through the audit of Chinese Clinical Trial Registry (registration number: ChiCTR-COC-17013241). All study subjects provided informed consent prior to the inclusion of people in the study. The investigation conformed to the principles outlined in the Declaration of Helsinki.

### 2.3. Atrial Cardiomyocyte Culture

Primary neonatal atrial rat cardiomyocytes were isolated from 1–3-day-old Sprague-Dawley rats as described [21]. Briefly, neonatal rats were euthanized by decapitation, the atrium was dissected, minced, and digested with trypsin and collagenase, and the isolated cells were preplated twice for 60 min to eliminate fibroblasts. The nonadherent myocytes were then plated in plating medium containing 199 media supplemented with HEPES, MEM nonessential amino acids, glucose, glutamine, 10% foetal bovine serum, vitamin B12, penicillin, and streptomycin on fibronectin-coated plates. Following overnight culture, cells were washed, and fresh medium with 2% foetal calf serum was added.

### 2.4. Western Blotting

Proteins were size-fractionated on 8–12% sodium dodecyl sulphate-polyacrylamide gels and transferred to polyvinylidene difluoride membranes. Membranes were blocked by 5% nonfat dry milk (NFDM) in phosphate-buffered saline (PBS) and incubated for 1 h at room temperature (RT). Membranes were washed with PBS containing 0.5% Tween-20, incubated with primary antibodies overnight, and then incubated with horseradish peroxidase- (HRP-) conjugated secondary antibody for 1 h. Antibodies against atrial natriuretic peptide (ANP), brain natriuretic peptide (BNP), beta-myosin heavy chain (*β*-MHC), skeletal alpha-actin (SKA), MEF2, P-HDAC4 (S632), P-HDAC5 (S498), HDAC4, HDAC5, H3K27ac (anti-Histone H3K27), and H4ac (acetyl-Histone H4K5, 8, 12, 16) were purchased from Abcam (Cambridge, UK). Antibodies against P-HDAC5 (S259) and P-HDAC4 (S246) were purchased from Cell Signaling Technology (Mountain View, CA, USA). HRP-goat anti-rabbit IgG secondary antibodies were obtained from Saierbio Technology Inc. (Tianjin, China). The images were captured on a UVP BioImaging System, and GAPDH was used as an internal control.

### 2.5. Immunofluorescence

Cultured atrial cardiomyocytes were washed with PBS and fixed with 4% paraformaldehyde for 30 min. After 3 washes with PBS for 5 min each, permeabilization of cell membranes was accomplished by applying 0.1% triton X in 0.5% NFDM supplemented with 1% foetal calf serum in PBS for 30 min at RT. Permeabilized cells were incubated with rabbit anti-*α*-actin, HDAC4, or HDAC5 antibody (1 : 800) diluted in 0.1% triton X, 1% NFDM, and 1.4% normal calf serum in PBS overnight at 4°C. Primary antibodies were withdrawn the next day, and cells were washed twice with 1X PBS for 5 min at RT. Secondary antibody FITC- or TRITC-labelled goat anti-rabbit was diluted (1 : 1,000) in the same primary antibody solution and applied to the cells for 1 h at RT. Cells were washed twice (1X PBS) and visualized and imaged using the ECLIPSE Ts2-FL fluorescence microscopy (Nikon, Tokyo, Japan).

### 2.6. Chromatin Immunoprecipitation (ChIP)

ChIP was performed according to the manufacturer's instructions. Briefly, atrial cardiomyocytes were fixed with 1% formaldehyde for 10 min at 37°C. Chromatin was sonicated, yielding DNA fragments of 200–800 bp. After preclearing with protein A/G agarose at 4°C for 1 h, samples were incubated with 10 *μ*g HDAC4, HDAC5, MEF2, H3K27ac, or H4ac antibody or IgG (as a control) with rotation at 4°C overnight. The cross-linking was reversed by incubation in 5 M NaCl/proteinase K solution at 65°C for 2 h. Precipitated DNA was purified using spin columns and subjected to polymerase chain reaction (PCR) analysis. Real-time PCR was performed using iQ SYBR Green Supermix and the iCycler real-time PCR detection system (Bio-Rad). The reaction conditions were as follows: denaturation at 95°C for 10 min, followed by 40 cycles of amplification and quantification at 95°C for 30 s, 60°C for 30 s, and 72°C for 1 min. The conditions of the melting curve analysis were as follows: 95°C for 15 s, 60°C for 15 s, and 95°C for 15 s. The primers used for PCR to identify the *ANP* and *BNP* promoter-binding sequence were as follows: *ANP* forward-5′CGT TGC CAG GGA GAA GGA3′, reverse-5′CAT TCT GTC ACT TGC GGC G3′; *BNP* forward-5′GCT CAG CAG GCA GGA ATG3′, reverse-5′TAG CCT CTC AGC AAC GGT G3′.

### 2.7. ELISA Assay

Frozen heart tissue samples were weighed, homogenized using an electric homogenizer on ice in PBS, and centrifuged at 10,000 g for 20 min at 4°C. The supernatant was used for subsequent ELISA analyses. AngII levels were measured in a 96-well plate by a sandwich ELISA method using a kit from Elabscience (Houston, TX, USA). For the assay, 100 *μ*L of standard and sample was added to wells that were coated with antibodies before incubation. The final concentrations were calculated by interpolation from standard curves according to the manufacturer's instructions.

### 2.8. Construction of Recombinant Adenovirus

The full-length DNAs of the *HDAC4* and *HDAC4*-mut (S246A, S632A) genes with BglII and XbaI cleavage sites and *HDAC5* and *HDAC5*-mut (S259A, S498A) genes with added KpnI and HindIII sites were synthesized by Genewiz (South Plainfield, NJ, USA) and ligated with the adenovirus shuttle plasmid pAdTrack-CMV (Stratagene, La Jolla, CA.). These constructs were then linearized with PmeI and homologously recombined in AdEasier-1 cells, a derivative of BJ5183 bacteria already containing the adenovirus backbone plasmid pAdEasy-1 (Stratagene/Agilent Technologies, Santa Clara, CA, USA). Positive clones were selected for culture, plasmid extraction, and PacI digestion. The larger fragment was recovered using a gel extraction kit and transfected into HEK293 cells via liposomes (Lipofectamine™ 2000; Invitrogen, Carlsbad, CA). After 8 or 10 days, the recombinant adenovirus was collected by repeated freezing and thawing of the HEK293 cells and used to infect HEK293 cells; after 2 or 3 days, the cells exhibited cytopathic effect, and the virus was collected. The TCID50 method was used to calculate the adenovirus titre. Subsequently, cardiomyocytes were infected using a multiplicity of infection of 50.

### 2.9. RNA-Seq

Total RNA from cell and heart tissue samples was extracted using a TRIzol reagent (Invitrogen, Carlsbad, CA, USA) following the manufacturer's instructions. Genome-wide rat gene expression profiling was performed using RNA deep sequencing by Annoroad Gene Technology Co., Ltd. (Beijing, China). Library construction was performed following the manufacturer's instructions provided by Illumina (San Diego, CA, USA). Samples were sequenced on an Illumina HiSeq 4000 instrument. Clean data were used in further analyses. Tophat2 [22] was used to map clean reads to the genome of rn5. Differentially expressed genes (DEGs) were identified using HTSeq [23] and edgeR package [24]. A fold change > 1.5 and false discovery rate (FDR) < 0.05 were considered significant. Finally, a heatmap was generated in the R language.

### 2.10. Statistical Analysis

Data are expressed as means ± SD. An unpaired Student's *t* test was used for statistical comparison between two groups after the demonstration of homogeneity of variance with an *F* test, and one-way ANOVA was used for comparison of more than two groups. A value of *P* < 0.05 was considered statistically significant.

## 3. Results

### 3.1. Patients with AF Manifest Increased Susceptibility to Hypertrophy and Display Atrial Hypertrophy

The clinical characters of the study subjects are shown in Table 1. The AF group exhibited greater mean atrial dimensions than the SR group, suggesting atrial hypertrophy in patients with AF. As AngII constitutes a major effector peptide of RAS, which contributes to cardiac hypertrophy pathogenesis [25]. We measured the atrial tissue AngII concentration to investigate the status of RAS. Atrial tissue AngII concentration was significantly elevated (Figure 1(a)), which indicated the activation of RAS in patients with AF and suggested that the environment of atrial tissue itself in these patients may stimulate cardiomyocyte hypertrophy. To determine the presence of the foetal gene expression program associated with cardiac hypertrophy [8, 9], we quantified the products of hypertrophy-related genes ANP and BNP in the atrial tissue of AF and SR groups. An increase in ANP and BNP protein expression was detected in the AF compared to SR atrial samples (Figure 1(b)).

### 3.2. Atrial Tissue in Patients with AF Exhibits Epigenetic Characteristics Permissive for Hypertrophy-Related Gene Transcription

Among the intracellular pathways that integrate mechanical and hormonal signals, MEF2 plays prominent regulatory roles in cardiac hypertrophy and remodelling [26, 27]. Atrial samples from patients with AF showed greater enrichment of MEF2 bound to the promoters of hypertrophy-related genes ANP and BNP than that in SR samples (Figure 2). Class II HDAC isoforms, such as HDAC4 and HDAC5, act as signal-responsive repressors of nuclear MEF2 activity in cardiac myocytes, with their spatial regulation providing a key mechanism for the neurohormonal control of such activity [28, 29]. We observed decreased chromatin-bound HDAC4 and HDAC5 on both *ANP* and *BNP* promoters (Figures 2(a) and 2(b)), indicating a permissive state for histone acetylation in atrial tissue from patients with AF compared to SR.

To further explore tissue-specific histone modification patterns in AF and SR, we analyzed the H3K27ac and H4ac enrichment in the promoters of these hypertrophy-related genes. ChIP assays demonstrated an enhanced H3K27ac and H4ac enrichment on promoters of *ANP* and *BNP* in atrial tissues from patients with AF compared to SR (Figures 2(a) and 2(b)). Together, these findings indicated an increased profile of epigenetic characteristics permissive for hypertrophy-related gene transcription in AF, consistent with increased susceptibility to hypertrophy.

### 3.3. AngII Induces Hypertrophy of Atrial Cardiomyocytes

At the cellular level, hypertrophy is accompanied by an increase in cardiomyocyte size and reinduction of a foetal cardiac gene program that ultimately weakens cardiac performance [30, 31]. Thus, the reinduction of foetal genes (encoding ANP, BNP, *β*-MHC, and SKA) is employed as a marker of hypertrophy [32]. Incubation with AngII resulted in an increase in the cell cross-sectional area of atrial cardiomyocytes (Figure 3(a)). AngII-treated cardiomyocytes also showed significantly increased level of proteins encoded by hypertrophy-related genes compared with the control (Figure 3(b)). Conversely, the AngII-induced atrial cardiomyocyte hypertrophy and hypertrophy-related gene reactivation could be alleviated by ARB losartan (100 *μ*mol/L; Merck Sharp & Dohme Corp., Cramlington, UK).

### 3.4. AngII Induces HDAC4 and HDAC5 Phosphorylation and Nuclear Export

Numerous extracellular agonists and, in particular, those that act through G-protein-coupled receptors, such as adrenergic agonists, endothelin, and angiotensin, promote cardiomyocyte hypertrophy by modulating the activities of chromatin remodelling enzymes, which act as global regulators of the cardiac genome during pathological remodelling of the heart [33–35]. However, class II HDAC levels do not change in stressed myocardium [36]. Instead, these HDACs are shuttled from the nucleus to the cytoplasm in response to stress signals, suggesting a posttranslational mechanism to cardiac growth repression [19]. We found that HDAC4 and HDAC5 were located in the nucleus in approximately 90% of atrial cardiomyocytes under basal conditions. In contrast, AngII incubation caused HDAC4 and HDAC5 to translocalize and accumulate in the cytosol (Figures 4(a) and 4(b)), although total protein levels did not appear to change.

Class II HDACs share high structural homology in the region surrounding the phosphorylation sites in their N-terminal domains which contain docking sites for 14-3-3 proteins. Phosphorylation of their signal-responsive serine results in their nuclear exclusion in a 14-3-3 protein-dependent manner [37–39]. AngII incubation increased HDAC4 and HDAC5 phosphorylation on their signal-responsive serine sites (Figure 4(c)), suggesting that AngII may phosphorylate HDAC4 and HDAC5 to induce their nuclear exportation and cytoplasmic accumulation.

### 3.5. AngII Increases Chromatin Acetylation and MEF2 Enrichment on Hypertrophy-Related Gene Promoters by Excluding HDAC4 and HDAC5

We next tested whether AngII-induced nuclear export of class II HDACs would inhibit the binding of class II HDACs to the promoter region of hypertrophy-related genes. The ChIP assay showed that AngII decreased HDAC4 and HDAC5 binding in the promoter region of hypertrophy-related genes (Figure 5). The functional bridge connection between chromatin modifiers and signalling mediators is established through transcription factors [40] such as MEF2, which is found in many protein complexes that are involved in gene activation under pathological conditions by modifying histones [41, 42]. As class II HDACs form a complex with MEF2 resulting in repression of genes harbouring MEF2-promoter-binding sites [18, 43, 44], we tested the enrichment of MEF2 binding to the promoter region of hypertrophy-related genes. ChIP assay demonstrated that AngII treatment promoted MEF2 binding to the promoter region of hypertrophy-related genes, perhaps owing to AngII-induced nuclear export of class II HDACs and subsequent release of MEF2-promoter-binding sites.

HAT has also been shown to associate with the same domain of MEF2 that is also dominated by class II HDACs, although the interaction of MEF2 with HATs and HDACs is mutually exclusive [45]. We further found that AngII enhanced chromatin H4ac and H3K27ac modification levels on the MEF2-promoter-binding sites of hypertrophy-related genes, suggesting that AngII may facilitate MEF2 binding and acetylation of chromatin histones on the promoter of hypertrophy-related genes by excluding HDAC4 and HDAC5. This AngII-induced redistribution of HDACs empowers MEF2 and other transcriptional activators to approach and associate with HATs [20], resulting in increased histone acetylation of chromatin on local promoters and activation of downstream hypertrophy-related genes that promote hypertrophy of atrial cardiomyocytes.

### 3.6. AngII-Induced CaMKII/PKD Pathway Activation Results in HDAC4 and HDAC5 Nuclear Export

The kinase(s) that phosphorylate class II HDACs has become the focus of cardiac hypertrophy study because they coupled extracellular stimuli to the intracellular genome by governing class II HDAC nuclear localization and function. CaM kinases and protein kinase D (PKD) have been implicated in hypertrophy and heart failure in rodents and humans [46]. We hypothesized that CaMKII and PKD may delivery hypertrophic signals from the G-protein-coupled receptors of AngII to class II HDAC phosphorylation sites. Inhibition of CaMKII and PKD kinase function using the respective inhibitors KN93 (5 *μ*mol/L) and CID755673 (20 *μ*mol/L) partially prevented AngII-induced atrial cardiomyocyte hypertrophy and alleviated AngII-induced reexpression of hypertrophy-related genes (Figures 3(a) and 3(b)). CaMKII and PKD inhibitors could also decrease HDAC4 and HDAC5 phosphorylation and nuclear export (Figures 4(a) and 4(b)). These results suggested that AngII selectively targeted specific class II HDACs partially in a CaMKII- and PKD-dependent manner with consequent induction of atrial hypertrophy.

### 3.7. Class II HDAC Dephosphorylation Retards Their Nuclear Export and Antagonizes AngII-CaMKII/PKD-HDAC Signalling

Dephosphorylation of these sites antagonizes AngII-CaMKII/PKD-HDAC signalling, promoting class II HDAC nuclear retention. We mutated the serine phosphorylation sites of HDAC4 and HDAC5 and infected atrial cardiomyocytes with adenovirus harbouring mutated (lacking the three CaMKII/PKD phosphorylation sites) or wild-type (wt) versions of these proteins (Ad-mut-HDAC4, Ad-mut-DHAC5, Ad-HDAC4, or Ad-HDAC5) (Figure 6(a)). As expected, overexpression of Ad-HDAC4 and Ad-HDAC5 strongly repressed AngII-induced hypertrophy-related gene expression (Figures 6(b) and 6(c)), whereas HDAC4-mut and HDAC5-mut further strengthened the repression of AngII-induced hypertrophy-related gene expression (Figures 6(b) and 6(c)).

### 3.8. Atrial Energy Remodelling May Constitute an Upstream Influencer of Structural Remodelling

Mitochondrial energy dysfunction is also suggested as an atrial arrhythmogenic substrate [47, 48]. To assess the status of cardiac mitochondrial metabolism-related genes in AF, atrial cardiomyocytes were incubated with AngII for 48 h and subjected to RNA-Seq. Cardiac mitochondrial metabolism-related genes changed more extensively than cardiac structural genes under pathological hypertrophic conditions (Figure 7). Notably, these AngII-induced atrial energy remodelling changes could be reversed by the ARB losartan.

## 4. Discussion

### 4.1. Patients with Atrial Cardiomyopathy Display Atrial Hypertrophy

We have demonstrated that AngII-induced atrial structural remodelling plays an important role in the progression of AF [4, 5]. In 2016, the European Heart Rhythm Association postulated the concept of atrial cardiomyopathy, emphasizing the importance of atrial structural remodelling in AF pathogenesis. In the present study, a comparison of the clinical echocardiography materials of patients with AF or SR showed that the atrial diameter and the levels of proteins encoded by hypertrophy-related genes were much greater in the former, indicative of atrial hypertrophy in AF. These results were also consistent with the histopathologically characterized cardiomyocyte hypertrophy in EHRAS class I and III atrial cardiomyopathy [5].

### 4.2. Atrial Hypertrophy Promotes the Progression of Atrial Electrical and Functional Remodelling

The newly proposed atrial cardiomyopathy definitions highlight the tight relationship between structural, electrophysiological, and functional remodelling in atrial pathogenic substrates. Atrial hypertrophy, the major component of atrial structural remodelling, causes conduction abnormalities, wavelength shortening, and increased AF [49]. These are also observed following prenatal corticosteroid exposure-induced hypertension and atrial hypertrophy in sheep [50]. Specifically, hypertension induces progressive atrial hypertrophy, which prolongs atrial refractoriness and slows conduction, promoting the occurrence of AF [51].

The atria significantly contribute to cardiac function [52, 53]. In addition to their impact on ventricular filling, they serve as a volume reservoir for pulmonary vein (PV), as a return to modulate left ventricular (LV) filling and cardiovascular performance during LV systole, as a conduit for PV return during early LV diastole, and as a booster pump that augments LV filling during late LV diastole [5]. Long-term maladaptive atrial hypertrophy results in enlarged atrial volume and impaired atrial mechanical function. Hypertension-induced atrial hypertrophy reduces the left atrial emptying fraction [49], with atrial hypertrophy-induced left atrial dilation also contributing to a loss of atrial mechanical function, which in turn leads to disability [54]. Thus, increased atrial volume may represent a marker of impaired atrial performance and daily activities in older individuals [54].

### 4.3. Nuclear Epigenetic Mechanisms Contribute to the Transcriptional Regulation of Atrial Hypertrophy

Emerging evidence suggests that epigenetic mechanisms are involved in cardiac remodelling [13]. We observed enhanced H3K27ac and H4ac enrichment in promoters of hypertrophy-related genes in atrial tissues from AF. The associated “loose” epigenetic environment would provide sufficient space for cardiac transcription factors to interact with promoter DNA sequences and favour the transcription of hypertrophy-related genes. We also investigated whether the acquisition of H3K27ac and H4ac might assist MEF2 binding to the promoters of the hypertrophy-related genes. Collectively, the data presented in Figure 5 suggest a model whereby the histone modification of H4ac and H3K27ac at the promoter may provide a loosen chromatin environment that is permissive for the recruitment of MEF2. Thus, H3K27ac and H4Ac facilitate a “relaxed” chromatin structure that provides accessible promoter DNA for recognition by MEF2, further facilitating its binding to promoters of hypertrophy-related genes.

Our results demonstrate that the hypertrophy stimulus AngII-induced exclusion of HDAC4 and HDAC5 from the hypertrophy-related gene promoter regions was accompanied by reversible increased enrichment of MEF2. We speculate that in physiological conditions, class II HDACs form a complex with MEF2 on gene regulatory elements harbouring MEF2-binding sites, resulting in gene repression. AngII-induced exclusion of HDAC4 and HDAC5 from the promoter regions released MEF2-binding sites, promoting MEF2-promoter-binding and facilitating the transcription of hypertrophy-related genes. The HAT P300 has also been shown to dock with the same domain of MEF2 that is occupied by class II HDACs [45]. Thus, MEF2 may act as a platform to respond to positive or negative transcriptional signals by exchanging HATs and class II HDACs.

Transcriptional repression by class II HDACs strongly depended on their subcellular shuttling. HDAC4, HDAC5, HDAC7, and HDAC9 were found to have three conserved serine sites at the N-terminal domain [55]. Phosphorylation of at least one of these cites permits the connection with the chaperone 14-3-3, exposing the C-terminal nuclear export signal [42] and inducing shuttling from the nucleus to the cytoplasm. The shuttling of HDAC4 and HDAC5 from the nucleus to cytoplasm mediated by AngII phosphorylation may contribute to the exclusion of HDAC4 and HDAC5 from the chromatin of hypertrophy-related gene promoter regions. HDAC-induced deacetylation of histones in nucleosomes induces chromatin condensation and gene transcription repression by preventing the binding of transcription factors such as MEF2 and other components of the transcriptional machinery to gene promoter and enhancer regions. Thus, the cytoplasm nucleus translocation of class II HDACs may constitute a novel epigenetic mechanism regulating the transcription of hypertrophy-related genes.

### 4.4. Cytoplasmic CaMKII/PKD Pathways Are Involved in the Transcriptional Regulation of Atrial Hypertrophy

Signalling pathways that target gene expression may be applied to regulate hypertrophy-related gene expression. PKD belongs to the CaMK superfamily, the members of which exhibit regulatory effects on class IIa HDACs [56]. HDAC5 was previously identified as a phosphorylation target of PKD [56]. Cardiac-specific deletion of PKD in turn leads to protection from prohypertrophic stimuli (e.g., pressure overload via transverse aortic constriction chronic *β* adrenergic stimulation with isoprenaline, chronic AngII stimulation) [57]. Unlike PKD, CaMKII selectively phosphorylates HDAC4, suggesting a role for HDAC4 in CaMKII-dependent gene expression. Adrenergic receptor agonists, AngII and endothelin enhance CaMKII activity via G-protein receptor signalling [58]. In particular, AngII-induced hypertrophy-related gene expression and nuclear export of HDAC4 and HDAC5 could be ameliorated by PKD and CaMKII inhibitors, suggesting that PKD and CaMKII may constitute the cytoplasmic pathways that regulate the hypertrophic progression of atrial cardiomyopathy.

### 4.5. Atrial Energy Remodelling May Serve as an Upstream Influencer of Atrial Structural Remodelling

Evidence also exists that mitochondrial energy dysfunction may also constitute an atrial arrhythmogenic substrate [47, 48]. Our RNA-Seq data showed that the quantity of cardiac energy metabolism genes such as mitochondrial transmembrane protein, components of mitochondrial respiratory chain complex, and adenosine triphosphate synthesis-coupled protein changed more significantly than cardiac genes in the early stage of AngII incubation (Figure 7). These energy genes are specifically expressed highly in the heart. The results of our study thus demonstrate a possible mechanistic link between early atrial mitochondrial energy remodelling and atrial structural remodelling. Atrial mitochondrial energy genes changed much earlier and more markedly than structural remodelling genes under the initial stage of the pathological condition, suggesting that atrial energy remodelling may serve as the earliest initiator that triggers all other atrial remodelling processes including structural, electrical, and functional remodelling. Atrial energy remodelling may in turn represent a potential upstream therapeutic target for inhibiting and reversing atrial structural, electrical, and functional remodelling. Notably, the AngII-induced atrial structural and energy remodelling effects and correlated epigenetic transcriptional regulation and activation of cytoplasmic pathways could be reversed by the ARB losartan, further confirming the therapeutic function of ARB in atrial cardiomyopathy.

## 5. Conclusion

Atrial cardiomyopathy plays a key role in the pathogenesis of atrial dysfunction, AF, and cardiogenic stroke. Our results suggest a novel arrhythmogenic mechanism whereby epigenetic control of chromatin structure may play an important role in the progression of atrial cardiomyopathy (Figure 8). AngII induces histone acetylation via the cytoplasmic-nuclear shuttling of HDACs, which might provide a promising therapeutic strategy for atrial cardiomyopathy. Moreover, our findings will also fundamentally advance the fields of atrial function and atrial arrhythmogenesis research.

## Figures and Tables

**Figure 1:** Tissue levels of AngII and levels of proteins encoded by hypertrophy-related genes *ANP* and *BNP* from right atrial appendages are higher in patients with atrial fibrillation (AF) than those with sinus rhythm (SR). (a) Tissue levels of AngII were measured by ELISA. (b) Tissue levels of ANP and BNP were measured by western blotting. *N* = 5 per group. Data are shown as the means ± SD. Statistical significance was determined by one-way ANOVA followed by the Bonferroni posttest. ^∗^*P* < 0.05 vs. the N group.

**Figure 2:** Identification the enrichment of MEF2, HDAC4, HDAC5, and histone modifications on the hypertrophy-related genes *ANF* and *BNP* in human atrial tissue from patients with atrial fibrillation (AF) or normal sinus rhythm (N). Quantitative ChIP analysis for MEF2, HDAC4, HDAC5, and H3K27ac and H4ac enrichment at the promoter of *ANP* (a) and *BNP* (b) from chromatin isolated from AF or N atrial tissue. Histone modifications H3K27ac and H4ac, which have been associated with activation of gene expression, were measured at *ANF* (a) and *BNP* (b) gene promoters by ChIP. *N* = 3 per group. Data are shown as the means ± SD, statistical significance was determined by one-way ANOVA followed by the Bonferroni posttest. ^∗^*P* < 0.05 vs. N group. All ChIP data are plotted as fold enrichment over equivalent amounts of input DNA, H3K27ac:H3 Lys27 acetylation, and H4ac:H4 Lys acetylation.

**Figure 3:** AngII-induced atrial cardiomyocyte hypertrophy. Atrial cardiomyocytes were stimulated with saline, AngII, AngII + losartan, AngII + the PKD inhibitor CID755673, or AngII + the CaMKII inhibitor KN93 for 48 h and subjected to immunofluorescence staining with antibody against *α*-actin. (a) Cell surface area of atrial cardiomyocytes treated with different stimuli was examined. The mean surface area of atrial cardiomyocytes after treatment was obtained from 200 atrial cardiomyocytes per sample. (b) Atrial cardiomyocyte extracts from different groups were subjected to western blotting using anti-ANP, BNP, SKA, and *β*-MHC antibodies. Data are plotted as fold enrichment over equivalent amounts of GAPDH. Data are shown as the means ± SD. ^∗^*P* < 0.05. *N* = 3 per group. Statistical significance was determined by one-way ANOVA followed by the Bonferroni posttest. Mock: saline, Ang + PKD:AngII + PKD inhibitor CID755673, and Ang + CaMKII:AngII + CaMKII inhibitor KN93.

**Figure 4:** Regulation of subcellular localization and phosphorylation of HDAC4 and HDAC5. Atrial cardiomyocytes were stimulated with saline, AngII, AngII + losartan, AngII + the PKD inhibitor CID755673, or AngII + the CaMKII inhibitor KN93 for 48 h. The 5 groups were subjected to immunofluorescence staining with an antibody against HDAC4 (a) or HDAC5 (b). The results of the quantitative analysis of the cytosol/total HDAC4 (a), HDAC5 (b) ratio at baseline and after stimulation are shown. (c) Atrial cardiomyocyte extracts from these groups were subjected to western blotting using anti-P-HDAC4 (S246), P-HDAC5 (259), HDAC4, P-HDAC5 (S498), or HDAC5 antibodies. Data are plotted as fold enrichment over equivalent amounts of *β*-tubulin and are shown as the means ± SD. ^∗^*P* < 0.05. *N* = 3 per group. Statistical significance was determined by one-way ANOVA followed by the Bonferroni posttest. Mock: saline, Ang + PKD:AngII + PKD inhibitor CID755673, and Ang + CaMKII:AngII + CaMKII inhibitor KN93.

**Figure 5:** AngII-induced changes in the enrichment of MEF2, HDAC 4, HDAC5, and histone modifications on the promoter of hypertrophy-related genes *ANP* and *BNP* in cultured atrial cardiomyocytes. Quantitative ChIP analysis for MEF2, HDAC4, HDAC5, and H3K27ac and H4ac enrichment at promoters of *ANP* and *BNP*. All ChIP data are plotted as fold enrichment over equivalent amounts of input DNA and are shown as the means ± SD. ^∗^*P* < 0.05. *N* = 3 per group. Statistical significance was determined by one-way ANOVA followed by the Bonferroni posttest.

**Figure 6:** Dephosphorylation of HDAC4 and HDAC5 retard their nuclear export and antagonize AngII-induced expression of ANP and BNP. Atrial cardiomyocytes were transduced with the indicated adenoviruses Ad-GFP, Ad-HDAC4-flag, Ad-mut-HDAC4- (S246A, S632A) flag, Ad-GFP, Ad-HDAC5-His, or Ad-mut-HDAC5- (S259A, S498A) His and were stimulated with saline, AngII, or AngII and losartan for 48 h and subjected to western blotting using anti-ANP (b) and BNP (c) antibodies. Data are plotted as fold enrichment over equivalent amounts of *β*-tubulin and are shown as the means ± SD. ^∗^*P* < 0.05. *N* = 3 per group. Statistical significance was determined by one-way ANOVA followed by the Bonferroni posttest.

**Figure 7:** Heatmap showing the significantly altered genes related to cardiac mitochondrial energy metabolism and cardiac structure in the three groups. Blue and red represent low and high expression, respectively. Log_10_FPKM values are shown.

**Figure 8:** Working model for HDAC4- and HDAC5-mediated hypertrophy in AngII-induced atrial cardiomyopathy. Atrial cardiomyocytes have lower level of HDAC4 and HDAC5 enrichment on the promoter of chromatin of hypertrophy-related genes. After AngII induction, HDAC4 and HDAC5 shuttled from the nucleus to the cytoplasm. This results in loose chromatin structure and transcriptional induction of hypertrophy-related genes via deacetylation of chromatin histone and activation of the transcription factor MEF2, subsequently causing atrial hypertrophy.

**Table 1:** Patient characteristics.

	Sex	Age (year)	Protopathy	LVEF (%)	LA (mm)	RA (mm)	LV (mm)	Hypertension	Diabetes mellitus	Drugs
Sinus rhythm (*n* = 7)	M	29	Bicuspid aortic valves	73.0	3.4	3.3	7.2	No	No	Diuretics
	F	62	Coronary heart disease	37.2	3.7	3.9	3.9	Yes	Yes	Diuretics, calcium-channel blockers; nitrates
	M	80	Coronary heart disease	44.6	3.9	4.3	5.0	Yes	No	Diuretics, nitrates
	M	70	Coronary heart disease	61.5	5.0		4.6	Yes	Yes	No
	F	76	Coronary heart disease	45.1	3.2		4.2	Yes	Yes	Nitrates
	F	57	Coronary heart disease	76.1	3.7		4.4	Yes	No	Calcium-channel blockers; nitrates
	M	52	Coronary heart disease	48.7	4.0	4.0	5.3	Yes	No	Nitrates
Mean ± SD	…	60.9 ± 17.3	…	44.8 ± 23.4	3.8 ± 0.6	3.9 ± 0.4	4.9 ± 1.1	…	…	…
AF (*n* = 8)	F	66	Mitral valve prolapse	79.4	6.4	5.3	6.2	Yes	No	Diuretics
	M	71	Mitral valve prolapse	61.2	5.8	6.5	5.7	Yes	No	Diuretics, nitrates
	M	56	Coronary heart disease	47.4	4.0	5.0	5.7	No	No	No
	M	51	Atrial septal defect	59	5.5	6.5	4.6	No	No	Diuretics
	F	64	Mitral stenosis	48.6	4.6	5.8	4.0	No	No	Diuretics
	M	77	Atrial fibrillation	51.8	5.1	5.7	6.1	Yes	Yes	Calcium-channel blockers; nitrates
	F	79	Coronary heart disease	68.3	4.0	5.4	4.8	No	Yes	Nitrates, diuretics
	F	54	Mitral regurgitation	50.7	5.1	5.0	5.7	No	Yes	Calcium-channel blockers; nitrates
Mean ± SD	…	64.8 ± 10.5	…	58.3 ± 11.1	5.1 ± 0.8^∗^	5.7 ± 0.6^∗^	5.4 ± 0.8	…	…	…

M: male; F: female; LVEF: left ventricular ejection fraction; LA: left atrium; RA: right atrium; LV: left ventricle; ^∗^*P* < 0.05 vs. the sinus rhythm.

## Data Availability

Data available on request: the first author Liuying Zheng can be contacted for data request. Her contact email is zhengliuyi27@163.com.
